# Effects of Acupuncture Combined with Rehabilitation on Chronic Pelvic Pain Syndrome in Females: A Meta-Analysis Running Head—Acupuncture Combined with Rehabilitation on Chronic Pelvic Pain

**DOI:** 10.1155/2022/8770510

**Published:** 2022-03-15

**Authors:** Jie Zheng, Xinsheng Lai, Weifeng Zhu, Yingjie Huang, Chuyun Chen, Jianqin Chen

**Affiliations:** ^1^College of Acupuncture & Moxibustion Rehabilitation Clinical Medical, Guangzhou University of Chinese Medicine, Guangzhou, Guangdong 510405, China; ^2^Department of Acupuncture and Moxibustion, The Affiliated TCM Hospital of Guangzhou Medical University, Guangzhou, Guangdong 510130, China; ^3^Lai Xinsheng Inheritance Studio, National Famous and Old Chinese Medicine Expert, Guangzhou, Guangdong 510405, China; ^4^Department of Dermatological, Integrated Traditional Chinese and Western Medicine Hospital of Southern Medical University, Guangzhou, Guangdong 510000, China

## Abstract

**Objective:**

To investigate the clinical efficacy of this combined treatment for chronic pelvic pain syndrome (CPPS) by meta-analysis.

**Methods:**

Relevant articles were retrieved from PubMed, CNKI, Wanfang Data, Web of Science, and Embase, including randomized controlled trials on acupuncture combined with rehabilitation for CPPS in females.

**Results:**

A total of 224 articles were retrieved in this study, and 14 studies were finally identified for inclusion. Among them, the treatment group was treated with acupuncture combined with pelvic floor rehabilitation therapy, while the control group was treated with acupuncture or pelvic floor rehabilitation therapy. Meta-analysis showed that the treatment effective rate in the treatment group was significantly higher than that in the control group (OR = 6.54; 95% CI: 4.20, 10.21; *P* < 0.05). After treatment, compared with the control group, the treatment group showed lower incidences of adverse reactions (OR = 0.16; 95% CI: 0.09, 0.27; *P* < 0.05), bladder prolapse (OR = 0.36; 95% CI: 0.18, 0.73; *P* < 0.05), cervical prolapse (OR = 0.22; 95% CI: 0.10, 0.49; *P* < 0.05), and pelvic peritoneal hernia (OR = 0.14; 95% CI: 0.05, 0.38; *P* < 0.05); in addition, the treatment group was also associated with lower pain score (SMD = −4.05; 95% CI: −6.75, −1.34; *P* < 0.05) and pelvic dysfunction score (SMD = -4.35; 95% CI: -5.37, -3.34; *P* < 0.05).

**Conclusion:**

Acupuncture combined with rehabilitation is effective for CPPS in females, which can significantly reduce the pain intensity and improve pelvic dysfunction of patients.

## 1. Introduction

Chronic pelvic pain syndrome (CPPS), by definition, is a common chronic pain syndrome that persists in the pelvis for more than 6 months or periodically attacks for more than 3 months [1]. This is a challenging disease for specialist physicians, which directly and seriously affects the health and quality of life of women [2]. However, the exact etiology and pathogenesis of CPPS remain unclear. Studies suggest that CPPS may overlap with dyspareunia and dysmenorrhea and gastrointestinal, genitourinary, neurological, endocrine, and musculoskeletal disorders; psychological and sociocultural factors may also responsible for CPPS [3, 4].

At present, CPPS is mainly treated with drugs and surgery [5, 6], but because CPPS is characterized by slow clinical onset, complex etiology, long duration, and recurrent attacks, the clinical efficacy of these two treatments is not satisfactory [7]. Acupuncture is also a commonly used treatment for CPPS; this treatment is to penetrate the needle into and stimulate specific parts of the human body using acupuncture manipulation such as lifting and thrusting, thus achieving a therapeutic effect [8]. According to a randomized controlled trial (RCT) by Qin et al. [9], the acupuncture group showed a higher efficacy than the sham acupuncture group in the treatment for chronic prostatitis/CPPS. Similarly, Lee et al. [10] also found that acupuncture was twice as effective as sham acupuncture for improving symptoms of chronic prostatitis/CPPS. However, the sample size of these studies is too small to determine whether acupuncture alone can achieve satisfactory efficacy. Rehabilitation therapy is a treatment plan developed for the recovery of pelvic floor function in women [11]. In recent years, a number of clinical studies in China have demonstrated that acupuncture combined with rehabilitation therapy will produce good clinical results in the treatment of CPPS in females [8, 12, 13]. However, the sample size of the individual studies on this combined treatment is small, and the results are not consistent across studies. Therefore, this meta-analysis aims to systematically analyze existing RCTs, thus providing evidence-based medical evidence for the further clinical use of acupuncture combined with rehabilitation therapy for CPSS in females.

## 2. Materials and Methods

### 2.1. Literature Retrieval

Relevant RCTs were searched from PubMed, CNKI, Wanfang Data, Web of Science, and Embase without time restrictions. The search terms were set as “chronic pelvic pain syndrome in females,” “acupuncture,” and “rehabilitation therapy”; the same kind of keywords were connected by “or” and different kinds of keywords by “and.”

### 2.2. Screening Criteria

Inclusion criteria (PICOS) [14]: (1) population: female patients diagnosed with CPPS, and their clinical data was complete; (2) intervention: patients in the treatment group were treated with acupuncture combined with pelvic floor rehabilitation therapy; (3) comparison: patients in the control group treated with acupuncture or pelvic floor rehabilitation therapy alone; (4) outcomes: including at least one of the following indicators: effective rate, incidence of adverse effects, incidence of bladder prolapse after treatment, incidence of cervical prolapse after treatment, incidence of pelvic peritoneal hernia after treatment, Visual Analogue Scale (VAS) score before and after treatment, and pelvic floor function before and after treatment; (5) studies: RCTs.

Exclusion criteria:(1) the literature included patients with tumors; (2) the study subjects were animals or cells; (3) the literature in which the data required by this meta-analysis were not provided and not available; the original text could not be obtained; the literature with too small sample size; (4) the literature with poor quality, missing data, and repeated reports; (5) case reports and systematic reviews; (6) non-RCTs; (7) incomplete clinical data; and (8) patients who are unwilling to participate in the study.

### 2.3. Data Extraction

Two evaluators independently screened literature and extracted data according to inclusion and exclusion criteria. The main extracted data included (1) basic characteristics of included studies; (2) basic information of patients; (3) sample size; (4) study design; and (5) outcome measures. Disagreements were resolved by discussion or consultation with a third evaluator. If necessary, the authors were contracted to consult the data not mentioned in the literature.

### 2.4. Literature Screening and Quality Evaluation

Literature screening process was as follows. First, the literature failing to meet the criteria was excluded by titles and abstracts. Then, through full-text reading, the literature with incomplete data or with evaluation indicator or study subjects inconsistent with the inclusion criteria were excluded. Finally, for the repeated reports or extending reports, the ones published recently or with complete data were included after rescreening.

### 2.5. Statistical Analysis

Stata 16.0 software was utilized for this meta-analysis. The chi-square test and I^2^ were used to access the heterogeneity among studies. A fixed-effect model was used when there was significant heterogeneity (I^2^ > 50% and *P* < 0.10). Otherwise, the random-effect model was adopted. Standard mean difference (SMD) was as an effect size for measurement data, while odds ratio (OR) and 95% confidence interval (CI) for categorical variables. Sensitivity analysis tests the stability of the overall results in the meta-analysis by ignoring the study alone. In addition, Begg funnel plots were used to determine the publication bias if the number of studies exceeded 10. *P* < 0.05 was considered to indicate a significant difference.

## 3. Results

### 3.1. Literature Retrieval Results

Totally 224 articles were retrieved based on the search strategy, and then 158 duplicates were excluded. Then, 42 articles were excluded by reading title/abstract, and 10 articles by reading the full text (7 with incomplete data and 3 with duplicate data). Finally, 14 studies were included [8, 12, 13, 15–25]. The screening process is shown in Figure 1, and the characteristics of each included study in Table 1.

### 3.2. Meta-Analysis of the Efficacy of Acupuncture Combined with Rehabilitation Therapy

Thirteen [8, 12, 13, 15–24] studies compared the efficiency of treatment between the groups. No significant heterogeneity was identified among these studies in the effective rate (I^2^ = 0.0%, *P* = 0.998), so the fixed-effect model was used for meta-analysis. The result showed that the effective rate of the treatment group was significantly higher than that of the control group (OR = 6.54; 95% CI: 4.20, 10.21; *P* < 0.05), Figure 2(a). In addition, the sensitivity analysis results (Figure 2(b)) showed that the new pooled results of the included studies did not change much, suggesting low sensitivity and a stable and reliable meta-analysis result. The funnel plot of the effective rate was in a symmetrical manner, indicating small publication bias of the 13 included, and a reliable meta-analysis result, Figure 2(c).

### 3.3. Meta-Analysis of the Incidence of Adverse Reactions and Pelvic Dysfunction

Nine articles [8, 12, 13, 15–20] compared the posttreatment incidence of adverse reactions, incidence of bladder prolapse, incidence of cervical prolapse, and incidence of pelvic peritoneal hernia between the two groups. No marked heterogeneity was found among these studies in the posttreatment incidences of adverse reactions (I^2^ = 0.0%, *P* = 0.972), bladder prolapse (I^2^ = 0.0%, *P* = 1.00), cervical prolapse after treatment (I^2^ = 0.0%, *P* = 0.978), and pelvic peritoneal hernia (I^2^ = 0.0%, *P* = 1.00), so a fixed-effect model was utilized for meta-analysis. The results showed (Figures 3(a)–3(d)) that compared with the control group, the treatment group has lower posttreatment incidences of adverse reactions (OR = 0.16; 95% CI: 0.09, 0.27; *P* < 0.05), bladder prolapse (OR = 0.36; 95% CI: 0.18, 0.73; *P* < 0.05), cervical prolapse (OR = 0.22; 95% CI: 0.10, 0.49; *P* < 0.05), and pelvic peritoneal hernia (OR = 0.14; 95% CI: 0.05, 0.38; *P* < 0.05). According to sensitivity analysis, the new pooled results did not change greatly after combining the effect sizes, suggesting low sensitivity and the stable and reliable meta-analysis results, Figures 4(a)–4(d).

### 3.4. Meta-Analysis of Pain and Pelvic Floor Dysfunction

Five articles [8, 13, 17, 18, 25] compared pain scores before and after treatment between the two groups. A fixed-effect model (I^2^ = 0.0%, *P* = 0.939) was used to analyze pretreatment pain scores before treatment, and the result showed no significant difference between the two groups (SMD = 0.04; 95% CI: -0.15, 0.23; *P* > 0.05), suggesting the comparability between the groups, Figure 5(a). By contrast, marked heterogeneity was found in posttreatment pain scores (I^2^ = 98.4%, *P* ≤ 0.001), so a random-effect model was employed for pooling the effect size; the result showed that the posttreatment pain scores of the treatment group after were significantly lower than that of the control group (SMD = -4.05; 95% CI: -6.75, -1.34; *P* < 0.05), Figure 5(b).

Five articles [8, 13, 21, 23, 24] compared pelvic floor dysfunction before and after treatment between the two groups. Before treatment, a fixed-effect model (I^2^ = 0.0%, *P* = 0.748) was required for meta-analysis; no significant difference was found in the score of pelvic floor dysfunction between the groups (SMD = -0.12; 95% CI: -0.29, 0.05; *P* > 0.05) Figure 5(c). After treatment, a random-effect model was utilized to combine the effect size (I^2^ = 89.40%, *P* ≤ 0.001); a markedly lower pelvic floor dysfunction score was in the treatment group compared with the control group (SMD = -4.35; 95% CI: -5.37, -3.34; *P* < 0.05), Figure 5(d).

Additionally, sensitivity analysis confirmed that the new pooled results did not change greatly after combining the effect sizes, suggesting low sensitivity and consequently the stable and reliable meta-analysis results, Figures 6(a)–6(d).

## 4. Discussion

CPPS is a syndrome with complex etiology and a long course of disease, seriously affecting the health and quality of life of patients. This syndrome is difficult to be diagnosed and treated, posing a challenge on clinicians. Therefore, CPPS, clinically, requires a treatment combining gynecology, surgery, internal medicine, rehabilitation, and psychology departments [26]. Current clinical studies have shown that the treatment for CPPS is difficult because the etiology of CPPS has not been clarified, which may be related to adenomyosis, endometriosis, and pelvic inflammatory disease [27, 28]. At present, although the diagnostic technique of CPPS is more mature, there is no exact treatment plan but many existing problems need to be solved urgently.

Acupuncture is one of vital therapeutic means of traditional Chinese medicine. For CPPS, acupuncture stimulates acupoints such as Guilai (ST29), Sanyinjiao (SP6), Zhongji (CV3), Guanyuan (CV4), and Zusanli (ST36), thereby dredging meridians, removing blood stasis, and improving blood circulation, and ultimately improving symptoms [29, 30]. Pelvic floor rehabilitation treatment requires spontaneous contraction of levator ani muscle, thus improving pelvic floor muscle strength and pelvic floor congestion. After the rehabilitation treatment, the abilities of the pelvic to anti-infection and to break up adhesions and soften scars are increased, and the exudation of inflammatory substances is reduced, thus facilitating the rapid absorption of effusion and relieving pain [17].

Acupuncture combined with pelvic floor rehabilitation therapy has been proved to significantly improve pelvic function to reduce the incidence of pelvic dysfunction, relieve pain, and eventually improve the quality of life of patients [31]. This result has confirmed that by contrast with one of the two treatments alone, the combination of the two can achieve better efficacy for CPPS. This meta-analysis here systematically analyzed the 14 included RCTs. We found that for CPPS, acupuncture combined with pelvic floor rehabilitation therapy significantly improved the effective rate and reduced the incidence of adverse reactions and complications such as bladder prolapse, cervical prolapse, and pelvic peritoneal hernia. In addition, this combined treatment decreases pain and pelvic floor dysfunction in CPPS patients. This is consistent with the results of existing studies. Huang et al. [15] showed that acupuncture combined with pelvic floor rehabilitation had a significant effect on female patients with CPPS and reduced pelvic dysfunction. Li et al. [17] found that for female patients with CPPS, acupuncture combined with pelvic floor rehabilitation effectively reduced the pain and improved pelvic dysfunction. Collectively, acupuncture combined with pelvic floor rehabilitation can achieve better efficacy for CPPS in females, which also decreases the incidence of adverse reactions and complications.

This study still has some limitations. First, all 14 studies included in this analysis are domestic ones. Based on the criteria for evaluation RCTs, the quality of these included articles is not very high, may leading to biases of the statistical results. Secondly, most of the included articles have no follow-up data and therefore cannot be scientifically evaluated for long-term efficacy of the treatment, thus reducing the reliability of the results. Additionally, the outcome measures of each article are recorded at different time points, resulting in time effect bias and thus causing certain interference with meta-analysis results. Third, this study mainly collects relevant articles by searching the electronic databases and by manual screening of included articles and their references, which may result in omissions due to possible shortcomings in the collection of the databases and search strategies.

## 5. Conclusion

In summary, for CPPS in females, acupuncture combined with pelvic floor rehabilitation can significantly improve effective rate, reduce the incidence of adverse reactions and complications, and decrease the pain and pelvic floor dysfunction of patients. It means that this combined treatment has a positive impact on the quality of life of CPPS. However, this conclusion still needs to be further verified by multicenter RCTs with high quality and large sample.

## Figures and Tables

**Figure 1:** Flow diagram of literature screening.

**Figure 2:** Meta-analysis of the effective rate of acupuncture combined with rehabilitation therapy for chronic pelvic pain syndrome (CPPS) patients. (a) Forest plot of effective rate; (b) sensitivity analysis of effective rate; (c) funnel plot of effective rate.

**Figure 3:** Forest plots of incidence of adverse reactions and pelvic dysfunction after acupuncture combined with rehabilitation therapy for CPPS. (a) Forest plot of incidence of total adverse reactions; (b) forest plot of incidence of bladder prolapse; (c) forest plot of incidence of cervical prolapse; (d) forest plot of incidence of pelvic peritoneal hernia.

**Figure 4:** Sensitivity analysis of incidence of adverse reactions and pelvic dysfunction after acupuncture combined with rehabilitation therapy for CPPS. (a) Sensitivity analysis of incidence of total adverse reactions; (b) sensitivity analysis of incidence of bladder prolapse; (c) sensitivity analysis of incidence of cervical prolapse; (d) sensitivity analysis of incidence of pelvic peritoneal hernia.

**Figure 5:** Meta-analysis of pain and pelvic floor dysfunction before and after acupuncture combined with rehabilitation therapy for CPPS. (a) Forest plot of pain scores before treatment; (b) forest plot of pain scores after treatment; (c) forest plot of pelvic floor dysfunction scores before treatment; (d) forest plot of pelvic floor dysfunction scores after treatment.

**Figure 6:** Sensitivity analysis of pain and pelvic floor dysfunction before and after acupuncture combined with rehabilitation therapy for CPPS. (a) Sensitivity analysis of pain scores before treatment; (b)sensitivity analysis of pain scores after treatment; (c) sensitivity analysis of pelvic floor dysfunction scores before treatment; (d) sensitivity analysis of pelvic floor dysfunction scores after treatment.

**Table 1:** Basic characteristics of the included studies.

Study	Year	Sample time	Cases treat/Con	Age (years)		Time of disease (years)		Study design	Outcome measures
				Treat group	Con group	Treat group	Con group		
He Langchi	2016	2012.02–2014.08	29/29	33.0 ± 1.2	32.1 ± 1.3	3.2 ± 0.1	3.4 ± 0.1	RCT	①②③④⑤
Chen Li	2017	2013.09–2016.12	43/43	33.5 ± 6.3	32.4 ± 5.7	2.4 ± 0.6	2.2 ± 0.5	RCT	①②③④⑤⑥⑦⑧⑨
Ye Minglong	2019	2017.08–2018.12	43/43	45.2 ± 7.0	44.3 ± 6.4	NR	NR	RCT	⑥⑦
Huang Jin	2019	2017.01–2018.09	42/41	31.8 ± 6.9	31.4 ± 7.0	2.2 ± 0.6	2.1 ± 0.6	RCT	①②③④⑤
Li Caiqiong	2019	2015.08–2018.12	86/86	33.5 ± 6.3	32.4 ± 5.7	2.4 ± 0.6	2.3 ± 0.5	RCT	①②③④⑤⑥⑦⑧⑨
Yang Haifeng	2016	2012.11–2016.12	40/40	32.1 ± 5.4	32.1 ± 6.0	3.2 ± 0.8	3.5 ± 0.9	RCT	①②③④⑤
Wang Lu	2016	2014.03–2015.12	60/60	30.4 ± 3.1	29.5 ± 2.1	NR	NR	RCT	①⑧⑨
Li Xing	2017	2018.05–2019.12	25/25	35.2 ± 1.2	35.1 ± 1.3	2.0 ± 0.3	2.4 ± 0.3	RCT	①②③④⑤⑥⑦
Li Feng	2021	2019.10–2020.12	15/15	37.5 ± 3.3	37.2 ± 3.2	NR	NR	RCT	①②③④⑤⑥⑦
Yang Yuhuan	2020	2018.02–2019.12	40/40	32.5 ± 5.8	35.4 ± 5.7	NR	NR	RCT	①
Cui Li	2016	2015.03–2016.05	19/19	40–61	41–62	5.2 ± 0.8	5.3 ± 0.7	RCT	①⑧⑨
Hou Xingming	2017	2014.03–2016.03	36/36	32 ± 1.8	31 ± 1.3	4 ± 0.3	3 ± 0.8	RCT	①②③④⑤
Zhang Wen	2020	2018.11–2019.11	43/43	44.7 ± 3.9	44.5 ± 3.7	3.5 ± 0.8	3.2 ± 0.6	RCT	①②③④⑤
Wang Xiaoyan	2019	2017.01–2018.12	50/48	54.1 ± 6.1	53.3 ± 5.8	3.2 ± 0.9	3.9 ± 0.1	RCT	①⑧⑨

*Note.* Treat: treatment (acupuncture combined with pelvic floor rehabilitation therapy); Con: control (acupuncture or pelvic floor rehabilitation therapy); RCT: randomized controlled trial; NR: not reported; ① effective rate; ② incidence of adverse effects rate; ③ incidence of bladder prolapse after treatment; ④ incidence of cervical prolapse after treatment; ⑤ iIncidence of pelvic peritoneal hernia after treatment; ⑥ pain score before treatment; ⑦ pPain score after treatment; ⑧ pelvic floor function before treatment; ⑨ pelvic floor function after treatment.

## Data Availability

The data used to support the findings of this study are available from the corresponding author upon request.

## References

[1] Fall M., Baranowski A. P., Elneil S. (2010). EAU guidelines on chronic pelvic pain. *European Urology*.

[2] Gelbaya T. A., El-Halwagy H. E. (2001). Focus on primary care: Chronic pelvic pain in women. *Obstetrical and Gynecological Survey*.

[3] Butrick C. W. (2003). Interstitial cystitis and chronic pelvic pain: New insights in neuropathology, diagnosis, and treatment. *Clinical Obstetrics and Gynecology*.

[4] Wozniak S. (2016). Chronic pelvic pain. *Annals of Agricultural and Environmental Medicine*.

[5] Carey E. T., As-Sanie S. (2016). New developments in the pharmacotherapy of neuropathic chronic pelvic pain. *Future science OA*.

[6] Hoffman D. (2015). Central and peripheral pain generators in women with chronic pelvic pain: Patient centered assessment and treatment. *Current Rheumatology Reviews*.

[7] Ding J. L., Yang C. G. (2013). Progress in diagnosis and treatment of chronic pelvic pain. *Medical Recapitulate*.

[8] Li C. Q. (2019). Effect of pelvic floor rehabilitation therapy combined with acupuncture on gynecological chronic pelvic pain syndrome. *The Medical Forum*.

[9] Qin Z., Zang Z., Zhou K. (2018). Acupuncture for chronic prostatitis/chronic pelvic pain syndrome: A randomized, sham acupuncture controlled trial. *The Journal of Urology*.

[10] Lee S. W., Liong M. L., Yuen K. H. (2008). Acupuncture versus sham acupuncture for chronic prostatitis/chronic pelvic pain. *The American Journal of Medicine*.

[11] Cao Y., Fu Q. B., Si J. W., Hu N., Lv J. (2019). Effect of non-invasive pelvic floor muscle rehabilitation therapy on postpartum pelvic floor function recovery. *Shanghai Nursing*.

[12] He L. C., Huang L., Fan Y., Zhong Y. Z., Ren J. (2016). Effect of acupuncture combined with pelvic floor rehabilitation therapy on pelvic function in females patients with chronic pelvic pain syndrome. *Shenzhen Journal of Integrated Traditional Chinese and Western Medicine*.

[13] Chen L. (2017). Effect of acupuncture combined with pelvic floor rehabilitation therapy on chronic pelvic pain syndrome in females. *Journal of Minimally Invasive Medicine*.

[14] Ghaffari M., Rakhshanderou S., Ramezankhani A., Noroozi M., Armoon B. (2018). Oral health education and promotion programmes: Meta-analysis of 17-year intervention. *International Journal of Dental Hygiene*.

[15] Huang J., Zhang Y. N. (2020). Effect of acupuncture combined with pelvic floor rehabilitation therapy on chronic pelvic pain syndrome in females. *The Medical Forum*.

[16] Yang H. F. (2019). 40 cases of chronic pelvic pain syndrome treated by acupuncture combined with pelvic floor rehabilitation therapy. *Hunan Journal of Traditional Chinese Medicine*.

[17] Li X. (2020). Observation of the effect of acupuncture combined with pelvic floor rehabilitation on chronic pelvic pain syndrome in females. *Health Guide*.

[18] Li F. (2021). Effect of acupuncture combined with pelvic floor rehabilitation therapy on chronic pelvic pain syndrome in females. *Fertility and Health*.

[19] Hou X. M., Shao X. (2017). The value of acupuncture combined with pelvic floor rehabilitation therapy in improving pelvic function in female patients with chronic pelvic pain syndrome. *Yiayao Qianyan*.

[20] Zhang W. (2020). Effect analysis of acupuncture combined with pelvic floor rehabilitation therapy on improving pelvic function in patients with gynecological chronic pelvic pain syndrome. *Reflexology and Rehabilitation Medicine*.

[21] Wang L. (2016). Clinical analysis of pelvic floor rehabilitation instrument combined with acupuncture at Huiyin point in the treatment of pelvic floor dysfunction in women. *Jilin Medical Journal*.

[22] Yang Y. H., Fu T. T. (2020). Effect of acupuncture combined with pelvic floor rehabilitation therapy on chronic pelvic pain syndrome in females. *Jia You Yun Bao*.

[23] Cui L., Li Y., Xu J. (2017). Effect of acupuncture combined with pelvic floor rehabilitation therapy on chronic pelvic pain syndrome in females. *The Medical Forum*.

[24] Wang X. Y. (2019). Clinical study of pelvic floor rehabilitation instrument combined with acupuncture at Huiyin point in the treatment of pelvic floor dysfunction in women. *China Health Care & Nutrition*.

[25] Ye M. L. (2019). The value of acupuncture and moxibustion combined with pelvic floor rehabilitation therapy in improving pelvic function of patients with chronic pelvic pain syndrome in gynecology. *China Reflexology*.

[26] Mitidieri A. M. d. S., Gurian M. B. F., Silva A. P. M. d. (2017). Effect of acupuncture on chronic pelvic pain secondary to abdominal myofascial syndrome not responsive to local anesthetic block: A pilot study. *Medical Acupuncture*.

[27] Wu J. M., Zhou Y. Y., Qin X. L. (2020). Pelvic-sacral tendon-regulation needling technique of acupuncture combined with manipulative reduction in treatment of postpartum pelvic girdle pain: A randomized controlled trial. *Chinese Acupuncture & Moxibustion*.

[28] Shen Z. Q., Chen F. X., Bai Y. N. (2018). Clinical effect of biofeedback therapy combined with electrical stimulation on chronic pelvic pain syndrome. *Chinese Journal of Family Planning*.

[29] Chen C. X., Wang C. X., Liu H. (2019). Clinical study of pelvic floor rehabilitation combined with drugs in the treatment of chronic pelvic pain. *Clinical Medical & Engineering*.

[30] Khan S. B., Khan B. K. (2019). Clinical study of pelvic floor rehabilitation combined with drugs in the treatment of chronic pelvic pain. *World Latest Medicine Information*.

[31] Mitidieri A. M. S., Baltazar M. C. D. V., da Silva A. P. M. (2020). Ashi acupuncture versus local anesthetic trigger point injections in the treatment of abdominal myofascial pain syndrome: A randomized clinical trial. *Pain Physician*.

